The article "Evidence for a Pro-Proliferative Feedback Loop in Prostate Cancer: The Role of Epac1 and COX-2-Dependent Pathways" was retracted in 2025. Reasons: duplicated images; overlap with earlier publications; unreliable data; unreliable results or conclusions.

# Evidence for a Pro-Proliferative Feedback Loop in Prostate Cancer: The Role of Epac1 and COX-2-Dependent Pathways

**DOI:** 10.1371/journal.pone.0063150

**Published:** 2013-04-30

**Authors:** Uma Kant Misra, Salvatore Vincent Pizzo

**Affiliations:** Department of Pathology, Duke University Medical Center, Durham, North Carolina, United States of America; Florida International University, United States of America

## Abstract

**Objective:**

In human prostate cancer cells, a selective Epac agonist, 8-CPT-2Me-cAMP, upregulates cell proliferation and survival via activation of Ras-MAPK and PI- 3-kinase-Akt-mTOR signaling cascades. Here we examine the role of inflammatory mediators in Epac1-induced cellular proliferation by determining the expression of the pro-inflammatory markers p-cPLA2, COX-2, and PGE_2_ in prostate cancer cells treated with 8-CPT-2Me-cAMP.

**Methods:**

We employed inhibitors of COX-2, mTORC1, and mTORC2 to probe cyclic AMP-dependent pathways in human prostate cancer cells. RNAi targeting Epac1, Raptor, and Rictor was also employed in these studies.

**Results:**

8-CPT-2Me-cAMP treatment caused a 2–2.5-fold increase of p-cPLA2^S505^, COX-2, and PGE_2_ levels in human prostate cancer cell lines. Pretreatment of cells with the COX-2 inhibitor SC-58125 or the EP4 antagonist AH-23848, or with an inhibitor of mTORC1 and mTORC2, Torin1, significantly reduced the Epac1-dependent increase of p-cPLA2 and COX-2, p-S6-kinase^T389^, and p-AKT^S473^. In addition, Epac1-induced protein and DNA synthesis were greatly reduced upon pretreatment of cells with either COX-2, EP4, or mTOR inhibitors. Transfection of prostate cancer cells with Epac1 dsRNA, Raptor dsRNA, or Rictor dsRNA profoundly reduced Epac1-dependent increases in p-cPLA2 and COX-2.

**Conclusion:**

We show that Epac1, a downstream effector of cAMP, functions as a pro-inflammatory modulator in prostate cancer cells and promotes cell proliferation and survival by upregulating Ras-MAPK, and PI 3-kinase-Akt-mTOR signaling.

## Introduction

Prostate cancer is the most commonly diagnosed malignancy of men [1]. Various factors promote the growth and progression of prostate cancer. There is a well known association between the acquisition of androgen-independent growth and a potentially greater likelihood of metastasis [2]. There is also growing evidence that inflammatory changes in prostate tumors may promote growth [3]–[8]. Approximately 15–20% of all cancer deaths worldwide are linked to infection and inflammation [9]. While these deaths may primarily be attributed to these processes, pathologic, molecular, and epidemiological studies support the hypothesis that chronic inflammation is linked to cancer progression [10]. The inflammatory microenvironment of tumors is characterized by the presence of host leukocytes both in the supporting stroma and tumor areas [11]. In addition, the tumor milieu contains inflammatory mediators such as chemokines, cytokines, reactive oxygen species, and prostaglandins [3]–[8]. Cancer development in the presence of chronic inflammation involves cyclooxygenase-2 (COX-2), and activation of several transcription factors including NFκB, STAT3, activator protein-1, and hypoxia inducible factor 1α [3]–[8].

Prostaglandins and leukotrienes are key modulators that mediate crosstalk between epithelial cells and their surrounding stromal cells [3]–[7]. Arachidonic acid (AA) is a major ingredient of animal fat and the biologically active lipids derived from this substrate have crucial roles in chronic inflammation and cancer. Upon cellular stimulation, AA is released from membrane phospholipids by p-cPLA2 and then converted to different prostaglandins (PGs) by specific enzymes [6], [12]. COX-2 is the inducible isoform of the rate limiting enzyme that converts AA to proinflammatory prostaglandins. Among these PGE_2_ plays a predominant role in promoting tumor growth. PGE_2_ elevates expression of the antiapoptotic protein Bcl2 and activates cAMP generation [13]. PGE_2_ increases Epac expression, Rap1 activation, and Akt phosphorylation [14], [15]. Under normal conditions, COX-2 expression is low or not detected in most tissues; however, its overexpression together with activation of cytosolic PLA2 by phosphorylation is a feature of inflammatory reactions [16]. Several signal transduction pathways regulate COX-2 gene expression including Ras-MAPK, PKA, and PKC [17]–[20]. Overexpression of COX-2 occurs in breast, lung, colon, and prostate cancers [3]–[8]. *In vitro*, human prostate cancer lines PC-3, DU145, and LnCap express COX-2 [6], [12]. Inhibition of COX-2 slows proliferation and/or upregulates apoptosis in both androgen-independent and dependent human prostate cancer cell cultures. Treatment of LnCap cells with the COX-2 inhibitor NS398 or celecoxib induces apoptosis and decreases expression of Bcl2, *in vivo,* and inhibition of Cox-2 suppresses the invasiveness of DU-145 and PC-3 cells [12]. Treatment of PC-3 tumor-bearing mice with NS-398 suppresses tumor cell proliferation and induces tumor regression [21]. An additional effect is that COX-2 inhibitors suppress upregulation of VEGF which is important for tumor angiogenesis [3]–[7], [12]. Inflammation-associated histological aggressiveness in prostate cancers correlates with an increase in PSA levels [22]. In clinical trials of prostate cancer patients, COX-2 inhibitors cause a decrease in prostate specific antigen (PSA) levels and tumor cell doubling time. In addition, COX-2 activation and increased levels of PGE_2_ occur in tumor patients [23]–[26]. PGE_2_ acts through four cell surface receptors known as EP1, EP2, EP3, and EP4 [27]-[31].

PGE_2_ receptors expressed by human prostate cancer lines are of the EP2 and EP4 subtypes [28]. Binding of PGE_2_ to EP2 is coupled to G proteins which activate adenylyl cyclase leading to an increase in intracellular cAMP. This activates kinases such as PKA, Epacs, PI 3-kinase, and GSKβ3. PGE_2_ increases EP2 receptor mRNA, increases cAMP levels, and enhances cell proliferation. Expression of EP2 and EP4 receptors is significantly increased during the progression of prostate cancer and ectopic expression of these receptors in LnCap cells enhances PSA production [32].

The mammalian target of rapamycin (mTOR) is a Ser/Thr kinase that integrates signals from external stimuli [33]–[39] regulates many processes including cell proliferation. mTOR exists in two distinct complexes, mTOR1 and mTORC2. Several recent studies demonstrate that PGE_2_ upregulates mTORC1 and mTORC2 signaling. For example, PGE_2_-mediated endothelial cell survival is regulated by mTORC2 [40]. PGE_2_-mediated chemotaxis and chemokine release from mast cells is regulated by mTORC2 activation and this is reduced by pretreatment of cells with the active site mTOR inhibitor Torin1 [41]. Moreover, inhibition of COX-2 and mTOR show direct and indirect anti-tumor effects in cancers, and both celecoxib and rapamycin cause significant tumor growth inhibition [42]. mTORC1 in addition to mTOR, contains the regulatory-associated protein of mTOR (Raptor), and a cluster of other regulatory proteins [33]–[39]. Raptor regulates the assembly of mTORC1, recruitment of kinase substrates, and subcellular localization of mTORC1. Akt activates mTORC1 by directly phosphorylating the TSC1/TSC2 complex thereby inhibiting its GAP activity and releasing GTP-bound Rheb to activate mTORC1 [33]–[39]. When activated, mTORC1 phosphorylates two main regulators of mRNA translation and ribosomal genesis, p70 S6-kinase (S6-kinase) and 4EBP1, thus stimulating protein synthesis [33]–[39]. The mTORC2 complex, in addition to mTOR, contains Raptor-independent companion of mTOR (Rictor) and other regulatory proteins. mTORC1 and mTORC2 phosphorylate different substrates to regulate distinct cellular functions. mTORC1 stimulates cell proliferation by increasing cap-dependent translation initiation which is mediated by its two major down stream targets S6 kinase and 4EBP. mTORC2 is insensitive to acute treatment with rapamycin and regulates many processes, including cell proliferation and survival, by phosphorylating kinases such as Akt, SG-kinase, and PKC [33]–[39]. Loss or inactivation of tumor suppressors such as p53, LKB1, PTEN, and TSC1/2, which antagonize PI 3-kinase-dependent activation of mTORC1, can promote tumorigenesis via increased signaling [33]–[39]. Increased levels and/or phosphorylation of downstream targets of mTORC1 occur in various human malignancies and correlate with aggressive tumor behavior and poor prognosis [33]–[39]. mTORC2 activity is necessary for development of prostate cancer caused by PTEN deletion [43].

cAMP regulates a wide range of processes including proliferation and apoptosis through the downstream effectors including PKA. The effect of cAMP is idiosyncratic and may either inhibit or stimulate cell proliferation in a PKA-dependent or PKA-independent manner [44], [45]. In cells where cAMP stimulates cell proliferation in a PKA-independent manner, cAMP activates Rap1 via Epac [45]–[48]. Here the effects of cAMP are mediated by PI 3-kinase/Akt signaling [45]–[48]. Treatment of prostate cancer cells with the Epac agonist 8-CPT-2Me-cAMP upregulates Epac1 expression, Rap1 activation, MAPK activation, Akt phosphorylation at T308 and S473 in a PI 3-kinase dependent and mTORC1 and mTORC2 activation as judged by phosphorylation of S6-kinase at T389, 4EBP1 at T37/36 and Akt at S473 residues, respectively [47], . Silencing Epac1 expression by RNAi or pretreatment with PI 3-kinase or mTOR inhibitors suppresses 8-CPT-2Me-cAMP-induced upregulation of Epac1 activation of MAPK, mTORC1, and mTORC2 signaling, and ultimately DNA and protein synthesis [47], [48]. Epac couples cAMP production to Rap1 and PI 3-kinase activation. Rap1, which is often elevated in highly metastatic prostate cancer cell lines, regulates signals involved in cell proliferation, survival, and metastasis [49]. Epac1 is upregulated after inflammation and plays a critical role in the activation of PKC-dependent PGE_2_ signaling via activation of Rap1 [50].

As reviewed above, chronic inflammation promotes tumor initiation, proliferation, and metastasis by upregulating the COX-2-PGE_2_-cAMP signaling cascade. 8-CPT-2Me-cAMP, a specific analogue of cAMP, binds to Epac1, but not PKA. In prostate cancer cells, this analog causes upregulation of Epac1, Rap1GTP, protein synthesis, DNA synthesis, and MAPK, and PI 3-kinase-Akt-mTORC1-mTORC2 signaling. As a consequence, protein and DNA synthesis are stimulated. These effects are down regulated by pretreatment of cells with inhibitors of MAPK, PI 3-kinase, mTORC1, or RNAis that target Epac1, Raptor, or Rictor [47], [48]. Here we consider the hypothesis that Epac1 functions as an inflammatory mediator in prostate cancer by promoting cell proliferation and survival. We investigated the regulation of the pro-inflammatory markers p-cPLA2, COX-2, and PGE_2_ in three human prostate cancer cell lines treated with 8-CPT-2Me-cAMP. Pretreatment of cells with COX-2 inhibitors, an mTORC1 and mTORC2 inhibitor, or transfection of cells with Epac1 dsRNA, Raptor dsRNA, or Rictor dsRNA down regulated 8-CPT-2Me-cAMP induction of p-cPLA2, and COX-2. Cancer cell proliferation was also suppressed. Thus whereas PGE_2_ regulates cAMP production and Epac-activation, Epac activation also results in COX-2-dependent PGE_2_ production. The net result is an autocrine-like cyclic process driving prostate cancer cell proliferation through upregulation of Ras-MAPK and PI 3-kinase-Akt-mTOR signaling.

## Materials and Methods

### Materials

Culture media were purchased from Invitrogen. 8-CPT-2Me-cAMP was purchased from Axxora LLC (San Diego, CA). Antibodies against mTOR, p-Akt^S473^, Akt1, S6-kinase, p-S6-kinase^T389^, p-cPLA2^Ser505^ and cPLA2 were purchased from Cell Signaling Technology (Beverly, MA). Antibodies against Epac1, COX-2, Raptor, Rictor, EP2, and EP4 were purchased from Santa Cruz Biotechnology (Santa Cruz, CA). Anti-actin antibodies were obtained from Sigma (St. Louis, MO). [^3^H]thymidine (specific activity 174 Ci/mmol and [^3^H]leucine (specific activity 115.4 Ci/mmol) were obtained from Perkin-Elmer Life Sciences. All other materials used were of analytical grade and were procured locally. COX-2 inhibitor SC-58125 or the EP4 antagonist AH23848 were purchased from Caymon (Ann Arbor, MI) and Torin1 was purchased from Tocris Biosciences (Minneapolis, MN).

### Human prostate cancer cell lines

In this study, we employed three human prostate cancer cell lines, 1-LN, DU145, and PC-3. As previously described [51], the highly metastatic 1-LN prostate cancer cell line was derived at this institution from a metastasis of the less metastatic PC-3 cells in nude mice and was a kind gift of Dr. Philip Walther (Duke University Medical Center, Durham, NC). These cells are available upon request. DU-145 and PC-3 cells were purchased from ATCC. They were grown in 6, 12, or 48 well plates in RPMI 1640 medium supplemented with 10% FBS, 2 mM glutamine, 12.5 units/ml penicillin, 6.5 μg/ml streptomycin and 10 nM insulin (RPMI-S) in an humidified CO_2_ incubator at 37°C. After reaching 90% confluency, the medium was aspirated and a fresh volume of RPMI-S medium added and the cells were used for the experiments described below.

### Qualitative PCR for COX-2, EP2, and EP4 in prostate cancer cells stimulated with 8-CPT-2Me-cAMP

1-LN, PC-3, and DU145 prostate cancer cells were grown as above. After reaching 90% confluency, the cells were washed twice with Hanks' balanced salt solution containing 10 mM HEPES, pH 7.4, and 3.5 mM NaHCO_3_ (HHBSS). A volume of fresh RPMI-S medium was then added and the cells were incubated for 5 min for temperature equilibrium. The cells were exposed to either buffer or 8-CPT-2Me-cAMP (100 μM) for 30 min and incubated as above. The reaction was terminated by aspirating the medium. Total RNA from the cells was extracted using RNeasy Minikits (QIAGEN, Valentia, CA) according to the manufacturer's instructions. RNA was quantified by absorbance at 260 nM. Total RNA was reverse transcribed with 1 μg of RNA in a 20-μl reaction, using Moloney murine leukemia virus reverse transcriptase (200 units) and oligo (dT) as the primer for 1 h at 40°C. The resulting cDNA (5 μg) was used as a template, and a 225-bp segment of the cDNAs of COX-2, EP2 and EP4 was amplified using a 20-mer upstream primers for (1) COX-2-forward; (5′-TGG TCT GGT GCC TGG TCT G -3′) and a COX-2-reverse (5′- AGT ATT AGC CTG CTT GTC TGG AAC -3′); (2) EP2-forward: (5′- TTC ATC CGG CAC GGG CGG ACC GC -3′) and EP2-reverse (5′- CCT CCT GAG AAA GAC AGT GCT -3′); and (3) EP4-forward: (5′- CCT CCT GAG AAA GAC AGT GCT -3′) and EP4-reverse (5′- AAG ACA CTC TCT GAG TCCT -3′). A 302-bp segment of mouse β-actin (constitutive internal control) cDNA was co-amplified using a set of primers provided in an R&D Systems kit (Minneapolis, MN). Amplification was performed in a Biometra 2:01 PM3 thermocycler for 28 cycles (one cycle:94°C for 45 s, 60°C for 45 s and 70°C for 45 s). PCR products were analyzed on a 1.2% agarose/ethedium bromide gel. The gels were photographed and the intensity COX-2, EP2, and EP4 mRNA and β-actin mRNA bands was quantified.

### Measurement of cPLA2, COX-2, Epac1, EP2, and EP4 expression in prostate cancer cells stimulated with 8-CPT-2Me-cAMP by Western blotting

Prostate cancer cells (3×10^6^ cells/well in 6-well plates) were incubated overnight in RPMI-S medium and washed twice with cold HHBSS. A volume of RPMI-S medium was then added to each well. After temperature equilibration, cells in the respective wells were exposed to either buffer or 8-CPT-2Me-cAMP (100 μM/30 min) and incubated as above. Reactions were stopped by aspirating the medium and a volume of lysis buffer, containing 50 mM Tris•HCl (pH 7.5), 120 mM NaCl, 1% nonidet P-40, 2.5 mM sodium fluoride, 1 mM sodium pyrophosphate, 0.1 mM sodium orthovanadate, 1 mM PMSF, 1 mM benzamidine, and leupeptin (20 μg/ml), over ice for 20 min. Cell lysates were scraped into new Eppendorf tubes and centrifuged for 5 min at 800×g at 4°C and the protein contents of lysates were determined. To equal amounts of lysate protein, a volume of 4x sample buffer was added and samples were boiled for 5 min. Samples were electrophoresed on 10% or 12.5% polyacrylamide gel, transferred to PDVF membrane, and immunoblotted for p-cPLA2S505, COX-2, Epac1, EP2, and EP4. Protein bands were detected and quantified by ECF and Phosphorimaging on a Storm 860 Phosphorimager. The respective membranes were reprobed for unphosphorylated target protein or actin. The specificity of the antibodies was determined by treating the cell with non-immune antibodies and cell lysates processed as above. Under the experimental conditions, no reactivity of these controls was observed.

### Measurement of PGE_2_ in prostate cancer cells stimulated with 8-CPT-2Me-cAMP

Prostate cancer cells (3×10^6^ cells/well in 6-well plates) were incubated overnight as above in RPMI-S medium and washed twice with cold HHBSS and a volume of RPMI-S medium was then added to each well. After temperature equilibration, cells in the respective wells were exposed to either buffer, or 8-CPT-2Me-cAMP (100 μM/30 min) and incubated as above. Reactions were stopped by aspirating the medium and a volume of lysis buffer was added on for 20 min. Cell lysates were scraped into new Eppendorf tubes and centrifuged for 5 min at 800×g at 4°C and the protein contents of the lysates were determined. PGE_2_ levels in cell lysates were determined with an ELISA kit (ENZO Life Sciences) according to the manufacturer's instructions.

### Measurement of protein synthesis in cancer cells stimulated with 8-CPT-2Me-cAMP

Prostate cancer cells (300×10^3^ cells/well in 48 well plates) were grown in RPMI-S in an humidified CO_2_ (5%) incubator at 37°C. At 90% confluency, the medium was aspirated and a volume of RPMI-S was added to the wells, followed by the addition of: (1) buffer; (2) 8-CPT-2Me-cAMP (100 μM/16 h); (3) (AH23848 1 μM/3 h); (4) AH23848 1 μM/3 h) then 8 CPT-2Me-cAMP; (5) SC58125 (1 μM/3 h); (6) SC58125 1 μM/3 h) then 8-CPT-2Me-cAMP; (7) Torin1 (250 nM/3 h); or (8) Torin1 (250 nM/3 h) then 8-CPT-2Me-cAMP. [^3^H] leucine (2 μCi/ml) was then added and the cells were incubated overnight as above. The reactions were terminated by aspirating the medium and monolayers were washed twice with ice-cold 5% TCA and the cells washed three times with ice-cold PBS. Cells were lysed in a volume of 1N NaOH (40°C 2 h), protein concentration was estimated and the lysates were counted in a liquid-scintillation counter [47], [48].

### Measurement of DNA synthesis in 1-LN cells stimulated with 8-CPT-2Me-cAMP

Prostate cancer cells (3×10^3^ cells/well in 48 well plates) were grown in RPMI-S) in an humidified CO_2_ (5%) incubator at 37°C. At 90% confluency, the medium was aspirated and a volume of RPMI-S was added, followed by the addition of compounds as described above. [^3^H] thymidine (2 μCi/ml) was then added and cells were incubated overnight. The reactions were terminated by aspirating the medium and cell monolayers were washed twice with ice-cold 5% TCA followed by three washings with ice-cold PBS. Cells were lysed in a volume of 1N NaOH (40°C/2 h), the protein concentration was estimated and the lysates were counted in a liquid scintillation counter [47], [48].

### Measurement of COX-2 or mTOR inhibitor effects on 8-CPT-2Me-cAMP induced-upregulation of p-CPLA_2_, and COX-2

Prostate cancer cells (3×10^6^ cells/6 well plates) incubated overnight in RPMI-S medium were washed twice with cold HHBSS and a volume of RPMI-S medium were added to each well. Cells in the respective wells were treated as described above. Reactions were stopped by aspirating the medium and a volume of lysis buffer was added on ice for 20 min. Cell lysates were scraped into Eppendorf tubes and centrifuged for 5 min at 800×g at 4°C and the protein contents of the lysates determined. The samples were then studied as described above.

### Measurement of COX-2 and mTOR inhibitor effects on 8-CPT-2Me-cAMP-induced-upregulation of p-S6-kinase^T389^ in Raptor immunoprecipitates of prostate cancer cells

Phosphorylation of S6-kinase at T389 is considered a measure of mTORC1 activation. Prostate cancer cells (3×10^6^ cells/well in 6-well plates) incubated overnight in RPMI-S medium were washed twice with cold HHBSS and a volume of RPMI-S medium was added to each well. Cells in respective wells were treated as described above. Reactions were stopped by aspirating the medium and adding a volume of CHAPS lysis buffer, containing 40 mM HEPES (pH 7.5), 120 mM NaCl, 1 mM EDTA, 10 mM sodium pyrophosphate, 10 mM β-glycerophosphate, 0.5 mM sodium orthovanadate, 0.3% CHAPS and Roche Protease inhibitor cocktail (1 tablet/10 ml). The cells were lysed on ice for 20 min. Cell lysates were scraped into new Eppendorf tubes and centrifuged for 5 min at 800×g at 4°C and then protein contents of the lysates was determined. Equal amounts of lysate protein (200–250 μg) were immunoprecipitated with Raptor antibodies (1:50) Santa Cruz Cat no. sc 81537), followed by the addition of 40 μl protein A agarose. The mixtures were incubated overnight with rotation at 4°C. Raptor immunoprecipitates were recovered by centrifugation (2000 rpm/5 min/4°C) and washed twice with cold CHAPS lysis buffer. A volume of 4× sample buffer was added to the samples which were then boiled for 5 min, centrifuged, electrophoresed (10% acrylamide gel), transferred to Hybond-P membrane. The membranes were immunoblotted with antibodies against p-S6-kinase^T389^. The protein bands were detected by ECF and quantified in a Storm^860^ Phosphorimager [47], [48].

### Measurement of mTORC2 activation by phosphorylation of Akt^S473^ in Rictor immunoprecipitates of cancer cells stimulated with 8-CPT-2Me-cAMP

Phosphorylation of Akt at S473 by Rictor is considered a measure of mTORC2 activity. Prostate cancer cells (3×10^6^ cells/well in 6-well plates) incubated overnight in RPMI-S medium were washed twice with cold HHBSS, and a volume of RPMI-S medium was added to each well. We investigated the effect of COX-2 inhibitors and the mTOR inhibitor Torin1 on phosphorylation of Akt^S473^ in Rictor immunoprecipitates of 1-LN cells under the conditions described above. The reactions were terminated by aspirating the medium and adding a volume of CHAPS lysis buffer (buffer B). The cells were lysed on ice for 15 min. Equal amounts of lysate protein (200–250 μg) were immunoprecipitated with anti-Rictor antibodies (1:50, Santa Cruz, CA, ca# 81538) by the addition of 40 μl of protein A agarose slurry. The contents were incubated with rotation overnight at 4°C. Rictor immunoprecipitates were washed with (1) lysis buffer B supplemented with 0.5 M NaCl; (2) lysis buffer B; and (3) Tris•HCl (pH 7.4) supplemented with 1 mM DTT, 1 mM PMSF, and 1 mM benzamidine by centrifugation at 2500 RPM for 5 min at 4°C. To Rictor immunoprecipitates a volume of 4× sample buffer was added, and the samples boiled for 5 min. After centrifuging, the supernatant was electrophoresed on polyacrylamide 10% gels, protein transferred to PVDF membrane and immunoblotted with antibodies against p-AKT^S473^. Protein bands were visualized and quantified by ECF and Phosphorimaging. The respective membranes were reprobed for Akt as the loading control [47], [48].

### The effects of Epac1 gene silencing on COX-2 expression in cancer cells stimulated with 8-CPT-2Me-cAMP

To determine the role of Epac1 in the activation of mTORC2 in prostate cancer cells treated with 8-CPT-2Me-cAMP, the expression of Epac1 was silenced by RNAi [47], [48]. The chemical synthesis of dsRNA homologous to the target Epac1 peptide sequence s204VAHLSN209 mRNA sequence 5′-TGT GGC CCA CCT CTC CAA CTC -3′ (Swiss Prot Epac1 primary accession number 0953958) was performed by Ambion (Austin, TX). dsRNAs were prepared by annealing the sense 5′- UGG CCC ACC UCU CCA ACU CU-3′ and antisense 5′- GAG UUG GAG AGG UGG GCA ACA -3′ and the annealed dsRNA strands were purified by an Ambion kit. Silencing Epac1 gene expression prior to stimulation with 8-CPT-2Me-cAMP was accomplished by transfection of cancer cells with 100 nM (48 h) of Epac1 dsRNA as described previously [47], [48]. Control cells were transfected with an equimolar concentration of scrambled RNA (Ambion Catalog number 4610) as above. The magnitude of Epac1 silencing in transfected cells, as measured by Epac1 mRNA and Epac1 protein levels, ranged between 60-65% [47], [48]. The cells in 6 well plates were treated as follows: (1) lipofectamine + buffer; (2) lipofectamine +8-CPT-2Me-cAMP (100 μM/30 min); (3) Epac1 dsRNA (100 nM/48 h) +8-CPT-2Me-cAMP (100 μM/30 min); or (4) scrambled dsRNA (100 nM/48 h) +8-CPT-2Me-cAMP (100 μM/30 min) and incubated as described above. The reactions were terminated by aspirating the medium, a volume of CHAPS lysis buffer B was added, the cells were then lysed on ice for 15 min, transferred to Eppendorf tubes, centrifuged (1000 RPM/5 min/4°C), and the supernatants transferred to new tubes and protein concentration determined. The samples were processed as described above.

### Measurement of the effects of silencing Raptor or Rictor RNAi silencing on the expression of p-cPLA2 and COX-2 in prostate cancer cells treated with 8-CPT-2Me-cAMP

Transfection of prostate cancer cells with Raptor dsRNA or Rictor dsRNA was performed as described below. To further ascertain the involvement of mTORC1 in 8-CPT-2Me-cAMP induced upregulation of S6-kinase, we silenced the expression of the Raptor gene by RNAi, which disrupts assembly of the mTORC1 complex and suppress phosphorylation of its downstream target S6-kinase. The annealed RNAi of Raptor was purchased from Sigma and consists of the sense sequent (5′-3′) UCU GCA AAG AUU UGU UGA GdT (ID# SAS1-16Hs01-00048387-AS). The cells were transfected with 100 nM annealed Raptor dsRNA and control cells were transfected with lipofectamine as described previously [47], [48]. Forty-eight h after transfection, the control cells were stimulated with either buffer, or 8-CPT-2Me-cAMP (100 μM/30 min/37°C). Cells for the negative control were transfected with scrambled dsRNA (100 nM/48 h, Ambion) and then stimulated with either buffer or 8-CPT-2Me-cAMP. The reactions were terminated by aspirating the medium and the cells were lysed in a volume of buffer B as described above. To equal amounts of lysate protein, a volume of 4× sample buffer added, samples boiled for 5 min, centrifuged and electrophoresed on 10% polyacrylamide gel. Proteins were transferred onto PVDF membranes and respective immunoblotted with anti-COX-2 and p-cPLA2 antibodies. Protein bands were visualized and quantified by ECF and phosphorimaging as described above. The samples were processed and studied as described above.

To confirm that 8-CPT-2Me-cAMP-induced activation of mTORC2 is involved in upregulation of cPLA2 and COX-2 we silenced Rictor gene expression by RNAi, which disrupts assembly of mTORC2 complexes and thus suppress mTORC2 activation. The siRNA probe was purchased from Ambion (small interfering RNA ID S226002) of the sense sequence (5′- GGG UUA GUU UAC AAU CAG C -3′) and antisense (5′- GCU GAU UGU AAA CUA ACC -3′). The cells were transfected with 100 nM of annealed Rictor dsRNA and control cells were transfected with lipofectamine as described previously [47], [48]. Forty-eight h after transfection, the control cells were stimulated with either buffer or 8-CPT-2Me-cAMP (100 μM/30 min/37°C). Cells for the negative controls were transfected with scrambled dsRNA (100 nM/48 h, Ambion) and then stimulated with either buffer or 8-CPT-2Me-cAMP as above. The reactions were terminated by aspirating the medium. The cells were lysed over ice for 20 min in CHAPS lysis buffer. The lysates were transferred to Eppendorf tubes, centrifuged at 800 RPM for 5 min at 4°C and the protein content of the supernatants was determined. To equal amounts of lysate protein, a volume of 4x sample buffer added, and the samples were boiled for 5 min, centrifuged, and electrophoresed on 10% polyacrylalmide gel. Proteins were transferred onto PVDF membranes and respective membranes immunoblotted with anti-p-cPLA2 or COX-2 antibodies. Protein bands were visualized and quantitated by ECF and Phosphorimaging.

## Results

### Upregulation of the inflammatory markers p-cPLA2, COX-2, PGE_2_, EP, and EP4 in prostate cancer cells stimulated with 8-CPT-2Me-cAMP

We first evaluated the pro-inflammatory environment in three androgen-independent human prostate cancer lines, namely, 1-LN, DU-145, and PC-3, by quantifying p-cPLA2^Ser505^, COX-2, EP2, EP4, and PGE_2_ in these cells stimulated with either buffer or 8-CPT-2Me-cAMP (Figure 1). Treatment of prostate cancer cells with 8-CPT-2Me-cAMP caused a 2-2.5-fold increase in the expression of p-cPLA2^Ser505^ compared to controls (Figure 1). A plausible mechanism by which Epac1 may activate cPLA2 is by elevating intracellular calcium and activating MAPKs. Epac1 regulation of Ca^2+^ release from the endoplasmic reticulum has been previously reported [52]. Epac1 increases intracellular Ca^2+^ by PLCγ-mediated hydrolysis of PIP2 generating IP3 which elevates intracellular Ca^2+^ [53]. All three prostate cancer lines stimulated with buffer showed negligible or very low levels of COX-2 mRNA and protein compared to 8-CPT-2Me-cAMP-stimulated cells which showed a 2-3-fold increase in COX-2 mRNA and protein (Figure 1A and B). Similar to COX-2, treatment of prostate cancer cells with 8-CPT-2Me-cAMP caused a 2-3-fold increase in intracellular PGE_2_ synthesis compared to controls (Figure 1C). Stimulation of prostate cancer cells with 8-CPT-2Me-cAMP also caused transcriptional and translational upregulation of EP2 and EP4 by 2-3-fold compared to controls (Figure 1A and B). Stimulation of 1-LN, DU-145, and PC-3 prostate cancer cells significantly upregulated Epac1 (Figure 1D).

**Figure 1:** 8-CPT-2Me-cAMP-induced expression of inflammation markers in prostate cancer cells. **Panel A**. Upregulation of COX-2, and EP2 and EP4 receptor mRNA in 1-LN, DU-145, and PC-3 prostate cancer cells stimulated with 8-CPT-2Me-cAMP (100 μM/30 min). The lanes are (1) buffer stimulated; and, (2) 8-CPT-2Me-cAMP-stimulated. **Panel B.** Immunoblot showing upregulation of p-cPLA2, COX-2, EP2, and EP4 in prostate cancer cells stimulated with 8-CPT-2Me-cAMP (100 μM/30 min). **Panel C.** A bar diagram showing 8-CPT-2Me-cAMP-induced upregulation of PGE_2_ synthesis in prostate cancer cells. Levels of PGE_2_ are expressed as pg PGE_2_/μg of cell protein. Values significantly different at 5% levels from buffer and treated cells are marked with an asterisk (*). **Panel D.** An immunoblot showing Epac1 protein levels in 1-LN and DU-145 and PC-3 prostate cancer cells stimulated with 8-CPT-2Me-cAMP(100 μM/30 min). Lanes in **Panel B, C, and D** are as in **Panel A**. All experiments were performed in triplicate and a representative immunoblot and the respective protein loading control actin or the unphosphorylated target proteins cPLA2 and Epac1 is shown.

### Inhibition of 8-CPT-2Me-cAMP-induced protein and DNA synthesis in prostate cancer cells by COX-2 and mTOR inhibitors

In the preceding section we demonstrated that Epac1 functions as a pro-inflammatory modulator in prostate cancer cells because it significantly elevated the expression of chronic inflammation markers (Figure 1). We have reported that 8-CPT-2Me-cAMP treatment of prostate cancer cells causes about a twofold increase in DNA and protein synthesis which is sensitive to LY-294002, rapamycin, or transfection with Epac1 dsRNA [47], [48]. To elucidate the involvement of chronic inflammatory signaling by PGE_2_ in 8-CPT-2-Me-cAMP-induced protein synthesis in 1-LN and DU-145 cells, we used the COX-2 inhibitor SC58125 (1 mM/3 h) (Figure 2A) or the EP4 antagonist AH32848 (1 mM/3 h). The role of mTOR in regulating 8-CPT-2Me-cAMP-induced protein synthesis was determined by pre-treating 1-LN cells with the mTOR inhibitor Torin1 (Figure 2B). In an identical fashion, we evaluated the role of PGE_2_ in 8-CPT-2Me-cAMP-induced DNA synthesis in 1-LN and DU-145 cells (Figure 3A), and of mTOR signaling on 8-CPT-2Me-cAMP-induced DNA synthesis in 1-LN cells (Figures 3B). Inhibition of PGE_2_-induced cAMP generation by the COX-2 inhibitor or EP4 antagonist significantly decreased inhibited 8-CPT-2Me-cAMP-induced protein (Figure 2A) and DNA synthesis (Figure 3A). Torin1 is an active site inhibitor of mTOR and similar to COX-2 inhibitors, pretreatment of cancer cells with Torin1 significantly inhibited the 8-CPT-2Me-cAMP-induced increase in protein (Figure 2B) and DNA synthesis (Figure 3B). These results support the role of Epac1 as a pro-inflammatory modulator in prostate cancer growth. They also suggest cross talk between COX-2-PGE_2_ and mTOR signaling cascades to promote cancer cell growth.

**Figure 2:** Suppression of 8-CPT-2Me-cAMP-induced protein synthesis in prostate cancer cells. **Panel A.** The bars in the diagram are: (1) buffer; (2) 8-CPT-2Me-cAMP (100 μM/16 h); (3) AH23848 (1 μM/3 h); (4) AH-23848 then 8-CPT-2Me-cAMP; (5) SC-58125 (1 μM/3 h) and (6) SC 58125 then 8-CPT-2Me-cAMP. The black bars in Panel A and B are data for 1-LN cells and the white bars in Panel A are data for DU-145 cells. **Panel B.** The bars in the diagram are: (1) buffer and 8-CPT-2Me-cAMP (100 μM/16 h); (3) Torin1 and (4) Torin1 then 8-CPT-2Me-cAMP. Protein synthesis as determined by quantifying the incorporation of [^3^H] leucine into cellular proteins is expressed as fmol [^3^H] leucine incorporated mg protein and is the mean ± SE from three separate experiments in each panel. Values significantly different for buffer versus inhibitor-treated cells (Figure 2A) and buffer versus Torin-treated cells (Figure 2B) at the 5% level are marked with an asterisk (*).

**Figure 3:** Inhibition of DNA synthesis by COX-2 (Panel A) and mTOR inhibitors (Panel B) in prostate cancer cells stimulated with 8-CPT-2Me-cAMP. The bars in **Panel A** and **B** are as in Figure 2. DNA synthesis as determined by quantifying the incorporation of [^3^H] thymidine into cellular DNA and is expressed as fmol [^3^H] thymidine incorporated mg protein and the data represent the mean ± SE from three independent experiments in each panel. Values significantly different from buffer and inhibitor-treated cells (Figure 3A) and from buffer and Torin1-treated cells (Figure 3B) at the 5% level are devoted by an asterisk (*).

### COX-2 inhibitors suppress 8-CPT-2Me-cAMP-induced increase in p-cPLA2 and COX-2

In Figure 1A, B we showed that stimulation of prostate cancer cells with 8-CPT-2Me-cAMP upregulated transcriptional and translational expression of COX-2 and p-cPLA2. In the next series of experiments, cells were treated with the COX-2 inhibitor or EP4 antagonist prior to exposure to 8-CPT-2Me-cAMP and effects on p-cPLA2 and COX-2 determined by Western blotting (Figure 4). These inhibitors significantly blocked the upregulation of p-cPLA2 and COX-2, further supporting the role of Epac1 as an inflammatory mediator in prostate cancer cell proliferation.

**Figure 4:** Suppression of elevated expression of the inflammation markers p-c-PLA_2_ and COX-2 in prostate cancer cells stimulated with 8-CPT-2Me-cAMP (100 μM/30 min by COX-2 inhibitors. A representative immunoblot of p-cPLA2 and COX-2 from three experiments along with their protein loading control is being shown. The lanes in p-cPLA2 and COX-2 immunoblots are: (1) buffer; (2) 8-CPT-2Me-cAMP (100 μM/30 min); (3) AH23848 (1 μM/3 h); (4) AH23848 then 8-CPT-2Me-cAMP (100 μM/30 min); (5) SC58125 (1 μM/3 h); (6) SC58125 then 8-CPT-2Me-cAMP (100 μM/30 min).

### COX-2 or the mTOR inhibitors block 8-CPT-2Me-cAMP-induced activation of S6-kinase in Raptor immunoprecipitates from prostate cancer cells

Pretreatment of cancer cells with the COX-2 inhibitor, the EP4 antagonist, or mTOR inhibitor, significantly inhibited 8-CPT-2Me-cAMP-induced protein synthesis (Figure 2A) consistent with the recent report that PGE_2_ regulates mTORC1 and mTORC2 signaling [42], [43]. S6-kinase and 4EBPs are direct downstream effectors of mTORC1 and play a central role in protein synthesis; therefore we employed Western blotting to evaluate activation of S6-kinase by phosphorylation (Figure 5). Incubation of cancer cells with 100 μM 8-CPT-2Me-cAMP for 30 min caused a 2-3-fold increase in p-S6-kinase^T389^ (Figure 5) showing significant activation of mTORC1 under these experimental conditions. Pretreatment of cells with both the COX-2 inhibitor, the EP4 antagonist, or the mTOR inhibitor markedly inhibited 8-CPT-2Me-cAMP-induced increase in p-S6-kinase^T389^ in Raptor immunoprecipitates (Figure 5A and B). As with the above studies, these results demonstrate cross talk between COX-2-PGE_2_ and mTORC1 signaling cascades in promoting prostate cancer cell proliferation.

**Figure 5:** Inhibition of 8-CPT-2Me-cAMP-induced activation of p-S6-kinase^T389^ in Raptor immunoprecipitates by COX-2 inhibitors (Panel A) or mTOR inhibitor Torin1 (Panel B) in prostate cancer cells. A representative immunoblot of p-S6-kinase^T389^ from three independent experiments are shown in **Panel A** and **Panel B**. The immunoblot lanes in **Panel A** are: (1) buffer; (2) 8-CPT-2Me-cAMP (100 μM/30 min); (3) AH23848 (1 μM/3 h); (4) AH23848 then 8-CPT-2Me-cAMP (100 μM/30 min); (5) SC 58125 (1 μM/3 h) and (6) SC58125 then 8-CPT (100 μM/30 min) and the lanes in **Panel B** are: (1) buffer; (2) 8-CPT-2Me-cAMP (100 μM/30 min); (3) Torin1 (250 nM μM/3 h) and (4) Torin1 than 8-CPT-2Me-cAMP.

### COX-2 inhibitors and Torin1 inhibit 8-CPT-2Me-cAMP-induced phosphorylation of Akt^S473^ in in Rictor immunoprecipitates from prostate cancer cells

PI 3-kinase activates Akt, a Ser/Thr kinase, which is the major downstream effector of the PI 3-kinase pathway and regulates cell survival, proliferation, and metabolism. Plasma membrane-bound Akt is phosphorylated at Thr308 in the catalytic domain by PDK1 and at Ser^473^ in the hydrophobic motif domain by mTORC2 [37]. Phosphorylation at both these positions is required for full activation of Akt1 [37]. Akt1 is also phosphorylated co-translationally at Thr^450^ in the turn motif by mTORC2 [54]. In an earlier report, we showed that stimulation of prostate cancer cells with 8-CPT-2Me-cAMP caused twofold increase in phosphorylation of Akt at Ser^473^ [47], [48]. This phosphorylation was sensitive to LY294002 and transfection with Rictor dsRNA and EPAC1 dsRNA, but was insensitive to acute rapamycin treatment. Pretreatment of cancer cells with the COX-2 inhibitor, EP4 antagonist or the mTOR inhibitor, significantly reduced the phosphorylation of Akt^S473^ in Rictor immunoprecipitates from 8-CPT-2Me-cAMP stimulated cells (Figure 6). This result suggests regulation of mTORC2 activation by COX-2.

**Figure 6:** Inhibition of 8-CPT-2Me-cAMP-induced activation of p-Akt^S473^ in Rictor immunoprecipitate by COX-2 inhibitors (Panel A) and a mTOR inhibitor (Panel B). A representative immunoblot of p-Akt^S473^ from three independent experiments are shown in **Panel A** and **Panel B**. The lanes in immunoblot in **Panel A** are: (1) buffer; (2) 8-CPT-2Me-cAMP (100 μM/30 min); (3) AH23848 (1 μM/3 h); (4) AH23848 then 8-CPT-2Me-cAMP (100 μM/30 min); (5) SC58125 (1 μM/3 h) and (6) SC58125 then 8-CPT-2Me-cAMP (100 μM/30 min) and the lanes in **Panel B** are: (1) buffer; (2) 8-CPT-2Me-cAMP (100 μM/30 min); (3) Torin (250 nM/3 h) and (4) Torin then 8-CPT-2Me-cAMP (100 μM/30 min).

### Transfection of prostate cancer cells with Epac1 dsRNA attenuates 8-CPT-2Me-cAMP-induced expression of COX-2

In our earlier reports, we have shown that silencing Epac1 expression by RNAi significantly suppresses proliferation of prostate cancer cells and down regulates the expression of signaling components of the MAPK and PI 3-kinase-Akt-mTOR signaling pathways [47], [48]. If Epac1 functions as an pro-inflammatory modulator in prostate cancer cells, then down regulating the expression of Epac1 by RNAi should inhibit the expression of COX-2. We demonstrate that silencing the expression of Epac1 nearly abolished 8-CPT-2Me-cAMP induced COX-2 expression in 1-LN prostate cancer cells (Figure 7), thereby identifying a mechanism by which PGE_2_-induced upregulation of COX-2 expression is mediated by Epac1 in an cyclic manner.

**Figure 7:** Effect of silencing Epac1 gene expression by RNAi on 8-CPT-2Me-cAMP-induced upregulation of COX-2 and Epac1 in prostate cancer cells. A representative immunoblot of COX-2 from three-independent experiments along with the protein loading control is shown. The lanes in COX-2 and Epac1 immunoblots of 1-LN and DU-145 cells are: (1) buffer + lipofectamine; (2) lipofectamine +8-CPT-2Me-cAMP (100 μM/30 min); (3) dsEpac1 RNA (100 nM/48 h) +8-CPT-2Me-cAMP (100 μM/30 min); and (4) scrambled dsRNA (100 nM/48 h) then 8-CPT-2Me-cAMP (100 μM/30 min).

### Effect of silencing Raptor or Rictor gene expression by RNAi on phosphorylation of cPLA_2_, and expression of COX-2 in prostate cancer cells stimulated with 8-CPT-2Me-cAMP

In an earlier report, we showed that Epac1 upregulates activation of MAPK, Akt, mTORC1 and mTORC2 in 1-LN prostate cancer cells [47], [48]. Silencing the expression of Epac1, Raptor and Rictor by RNAi profoundly attenuated the activation of these signaling cascades in prostate cancer cells treated with 8-CPT-2Me-cAMP [47], [48]. Silencing the expression of Epac1 by RNAi nearly abolished COX-2 expression in prostate cancer cells treated with 8-CPT-2Me-cAMP (Figure 7). Pretreatment of prostate cancer cells with the COX-2 inhibitor the EP4 antagonist, or the mTORC inhibitor significantly downregulated 8-CPT-2Me-cAMP-induced expression of p-cPLA_2_, COX-2, (Figure 4) S6-kinase^T389^ (Figure 5) and p-Akt^S473^ (Figure 6). This indicates that mTOR signaling is necessary for COX-2-mediated PGE_2_ signaling in prostate cancer cell lines. We therefore silenced the expression of Raptor and Rictor by RNAi and measured the expression of c-PLA2 and COX-2 in cells treated with 8-CPT-2Me-cAMP. Silencing the expression of Raptor and Rictor significantly downregulated by expression of both c-PLA2 and COX-2 (Figure 8). These results suggest a critical role of COX-2-mediated PGE_2_ synthesis and mTOR signaling in regulating 8-CPT-2Me-cAMP-induced growth and proliferation of prostate cancer cells in the inflammatory environment. Inhibition of 8-CPT-2Me-cAMP-induced upregulation of p-cPLA_2_ and COX-2 by Torin1 also suggest feed back regulation of inflammatory environment in prostate cancer cells by mTOR signaling.

**Figure 8:** Effect of RNAi silencing of Raptor or Rictor gene expression on 8-CPT-2Me-cAMP-induced increased expression of p-cPLA_2_ (Panel A) and COX-2 (Panel B) in 1-LN prostate cancer cells. – A representative immunoblot of p-cPLA2 (**Panel A**) and COX-2 (**Panel B**) from four experiments is shown. The lanes in the immunoblot in **Panel A** are: (1) lipofectamine + buffer; (2) lipofectamine +8-CPT-2Me-cAMP (100 μM/30 min); (3) dsRaptor RNA (100 nM/48 h) then 8-CPT-2Me-cAMP (100 μM/30 min); (4) dsRictor RNA (100 nM/48 h) then 8-CPT-2Me-cAMP (100 μM/30 min); (5) Rictor dsRNA (100 nM/48 h); (6) Torin (250 nM/3 h); (7) scrambled dsRNA (100 nM/48 h) then 8-CPT-2Me-cAMP (100 μM/30 min); and (8) Torin (250 nM/3 h) then 8-CPT-2Me-cAMP (100 μM/30 min). The lanes in the immunoblot in **Panel B** are: (1) lipofectamine + buffer; (2) lipofectamine +8-CPT-2Me-cAMP (100 μM/30 min); (3) Raptor dsRNA (100 nM/48 h); (4) Raptor dsRNA (100 nM/48 h) then 8-CPT-2Me-cAMP (100 μM/30 min); (5) Rictor dsRNA (100 nM/48 h) then 8-CPT-2Me-cAMP (100 μM/30 min); (6) Rictor dsRNA (100 nM/48 h); (7) scrambled dsRNA (100 nM/48 h) then 8-CPT-2Me-cAMP (100 μM/30 min); and (8) Torin1 (250 nM/3 h) then 8-CPT-2Me-cAMP (100 μM/30 min). The control is cPLA2 in Panel A and actin in Panel B. Also shown in **Panel C** are Raptor and Rictor protein levels in 1-LN cells transfected with Raptor dsRNA orRictor dsRNA. The lanes are as in Figure 7.

## Discussion

The role of inflammation in tumor progression is increasingly recognized as an important component of cancer cell growth [3]–[8]. The interplay of tumor cells, stromal elements, and inflammatory cells results in a complex milieu where host defense elements may actually promote tumor cell proliferation rather than killing. Therefore, a new view of cancer progression has emerged, which includes prostate malignancies. According to the injury and regeneration model for prostate neoplastic transformation, injury caused by pathogens or pro-inflammatory cytotoxic agents triggers proliferation of prostate glandular cells, leading to the appearance of epithelial lesions [3]. Co-incubation of PC-3 and LnCAP prostate cancer cell lines with peripheral blood mononuclear cells causes a concentration-dependent increase in secretion of the pro-inflammatory cytokine IL-6 by these cells [55]. Inactivation of PTEN is prevalent in prostate cancer [43] and its loss induces a selective upregulation of pro-inflammatory cytokine CXCL8 signaling that sustains the proliferation and survival of PTEN-deficient prostate epithelium [3]-[7]. In the present work, we examined this model.

The salient findings of the current study are: (1) stimulation of human prostate cancer cells with 8-CPT-2Me-cAMP significantly upregulated the expression of p-cPLA2 COX-2, PGE_2_, EP2, EP4, and Epac1; (2) a COX-2 inhibitor, EP4 antagonist, or the mTOR inhibitor significantly inhibit 8-CPT-2Me-cAMP-induced expression of p-cPLA2, COX-2, and protein and DNA synthesis in these cells; (3) these inhibitors significantly decrease the activation of mTORC1 as judged by phosphorylation of S6-kinase^T389^ and mTORC2 as judged by phosphorylation of Akt^S473^; (4) transfection of cells with Epac1 dsRNA nearly abolishes the expression of COX-2; and (5) transfection of prostate cancer cells with Raptor or Rictor dsRNA, significantly inhibits p-cPLA2 and COX-2 expression. These results are summarized in Figure 9.

**Figure 9:** A schematic representation of a cyclic autocrine feedback loop promoting human prostate cancer cell proliferation.

Our previous studies of Epac-mediated events in prostate cancer were in response to the observation that ligation of the α_2_-macroglobulin-proteinase (α_2_M*) cell surface signaling receptor, GRP78, results in activation of Gs-mediated cAMP production [56]. Given the role of cAMP in cellular regulation, we employed the cAMP agonist 8-CPT-2Me-cAMP to further elucidate the role of cAMP in prostate cancer proliferation [47], [48]. cAMP regulates a wide range of processes through the downstream effectors PKA, cyclic nucleotide-gated cation channels, and guanine nucleotide exchange factors involved in the regulation of Ras-related proteins. cAMP-dependent Epac activation drives pro-proliferative processes in many normal types as well as cancers including prostate cancer cells [47], [48], [56]–[60]. Epac1 is upregulated after inflammation and plays a critical role in the activation of PKC-dependent signaling by PGE_2_ via activation of Rap1 [50]. Activation of the Epac pathway also leads to many downstream signaling events including activation of mTORC1 and mTORC2 [47], [48]. Chronic activation of mTORC1 signaling is causally linked to liver damage and hepatocarcinoma [61]. By contrast, inhibition of mTORC1 and mTORC2 signaling attenuates prostate epithelial branching and invasion of surrounding mesenchyma [62].

The main catalytic functions of Epac are to activate Rap1 and Rap2 which are regulators of proliferation, migration, apoptosis, cytoskeleton restructuring, and inflammation [44], [45]. Epac-induced cell proliferation and anti-apoptotic signaling in prostate cancer cells is similar to that reported in cells treated with pro-inflammatory stimuli. This suggests a role for inflammation in Epac1-induced cell proliferation and survival observed in prostate cancer cells. Indeed, we found that Epac1 activation in prostate cancer cells upregulates expression of the pro-inflammatory markers, p-cPLA2, COX2, and PGE_2_. The mechanism(s) by which Epac1 functions in driving these pro-inflammatory signaling cascades in prostate cancer cells is not clear. One plausible mechanism is that in Epac1-stimulated cells, c-PLA2 activation generates AA, the substrate for COX-2 synthesis of PGE_2_. PGE_2_ binds to EP2/EP4 receptors generating cAMP, which binds to Epac1 and leads to Rap1 activation and activation of MAPK and PI 3-kinase-Akt-mTOR signaling. This is supported by studies with COX-2, PI 3-kinase, mTORC1, and mTORC2 inhibitors, which downregulate the expression of p-cPLA, COX-2, p-S6-kinase^T389^ and p-Akt^S473^. That Epac1 is directly involved in elevated COX-2 expression is also supported by observations of cells transfected with Epac1-dsRNA in which COX-2 expression is nearly abolished as well as activation of MAPK, PI-3-kinase-Akt-mTOR signaling, resulting in inhibition of cellular proliferation [47], [48].

Based on these results in human prostate cancer cell lines, we conclude that Epac1 functions as a pro-inflammatory mediator in prostate cancer cell proliferation and survival. These results help to explain at the mechanistic level observations made many years ago that α_2_M* binding to its then as yet unidentified signaling receptor resulted in cPLA2 [63], [64], COX-2 upregulation [65] and PGE_2_ generation [66], [67]. More recent studies establish the role of α_2_M* in activation of mTORC1 and mTORC2 which offers one explanation of why α_2_M activation, such as by PSA, drives pro-proliferative, anti-apoptotic, and pro-migratory signaling cascades [68]. In conclusion, we also hypothesize that in addition to COX-2 inhibitors, down regulation of EPAC1 is a promising therapeutic target in cancer management.
